# Rolling Bearing Fault Detection System and Experiment Based on Deep Learning

**DOI:** 10.1155/2022/8913859

**Published:** 2022-09-27

**Authors:** Bo Zhang

**Affiliations:** School of Network and Communication, Nanjing Vocational College of Information Technology, Nanjing 210023, China

## Abstract

The current situation of frequent small-scale accidents shows that the existing methods have not completely solved the problem of bearing failures, and new research methods need to be used to complete the study of bearing failures. To prevent the failure of rolling bearings and meet the need for timely detection of faults, this research is based on deep learning. Using the combination of deep transfer learning and metric learning methods, the identification and analysis of bearing multi-state vibration signals under different working conditions are carried out. The combination of SSAE-based similarity measurement criteria and deep transfer learning can reduce the differences between different domains. It is difficult to distinguish the data samples at the boundary and diagnose the problems that the physical meaning is difficult to understand. Through the bearing fault diagnosis analysis, the validity of the deep learning diagnosis model proposed in this paper is verified. The results show that the detection accuracy of the rolling bearing fault detection method based on LCM-SSAE is 0.6 percentage points higher than that of the rolling bearing fault detection method based on SSAE, which proves that the method is suitable for the fault detection of rolling bearing, and it also shows the effectiveness and robustness of the fault detection system of rolling bearing.

## 1. Introduction

The operating conditions of bearings have specific requirements, and the service life of rolling bearings is highly discrete and the service life cannot yet be precisely determined. It is possible to calculate a bearing's service life from the relevant bearing parameters. However, if service life is used as the evaluation standard, some bearings that are not defective will be treated as waste, resulting in waste. But it would also lead to the continued use of some defective bearings, reducing the accuracy of the equipment and even causing serious accidents. By detecting defects, it is possible to determine when to carry out maintenance and a maintenance plan. This reduces losses due to downtime caused by equipment failures and system maintenance costs and increases the efficiency and accuracy of the equipment. It is therefore very important to carry out fault detection on rolling bearings.

Scholars at home and abroad have conducted a lot of research on the fault diagnosis of rolling bearings. Xu and Hu proposed a new DS-ASR (DS-ASR) algorithm [1]. Cui et al. proposed a multi-scale morphological filtering algorithm based on the information entropy threshold (IET-MMF) [2]. Li et al. proposed a new signal processing method, that is multiscale morphological filtering (MMF) based on feature selection to detect row shaft bearings [3]. Xu et al. proposed a peak-based model decomposition method [4]. Pan and Yumei used LSTM neural network to identify the faults of rolling bearings [5]. Li et.al. referred to the idea of multilevel wavelet decomposition and adopts a new multilevel reconstruction filter to detect the early weak faults of rolling bearings [6]. Wang discussed bearing eigenfrequency analysis, smoothing to improve the signal-to-noise ratio [7]. Babiker et al. offered an integrated approach to fault diagnosis, combining backtracking strategies, advanced variation model decomposition (VMD), and infographics [8]. Gunerkar et al. proposed an accurate bearing fault diagnosis expert system [9]. Klausen et al. proposed a new multi-resonant region identification technique. This method combines computational order tracking with cepstral prewhitening in a new way to make the resonant frequencies in the signal emphasized [10]. These methods and systems cannot achieve the expected results and cannot provide timely early warning of failures, and deep learning can solve these problems well.

Deep learning can effectively improve the processing speed of data. He et al. introduced deep learning in the edge computing environment [11]. Ravi et al. proposed a new method based on deep learning [12]. Because these research materials are not complete and the research results are not perfect, they have not been accepted by the public and have not been promoted and used. The fault diagnosis of rolling bearings has the effect of filtering and processing data, and with deep learning, the efficiency of fault detection can be effectively improved. Therefore, this paper combines the above two factors, conducts experiments and provides some meaningful data.

In this paper, deep learning is combined with a rolling bearing defect detection system, and the following conclusions are drawn: to test the performance of ordered sparse autocoding, the ordered autocoding network is not used for feature extraction, but the softmax classifier is directly used for defect detection on the raw data. The softmax classifier is first trained on training samples and then its performance is tested on test samples. The overall percentage of correct responses is 70.571%.

## 2. Rolling Bearing Fault Detection System

Deep learning is a type of machine learning, and machine learning is the only way to realize artificial intelligence. Deep learning is a machine learning algorithm that can independently learn the properties of data. Since the technology was proposed in 2006, other countries have conducted relatively in-depth research into the technology. One of the most revealing studies is Google AlphaGo, whose excellent results have shocked the world. In contrast, Chinese research in this area has lagged somewhat behind, having started late. However, developments this year are still very optimistic. Many companies have launched their own spin-off products. Deep learning is the mapping of raw data from one space to another, which can also be understood as learning the features of the raw data. There are three categories of feature learning, each with its own development model and underlying idea. Supervised feature learning is the use of known category models to optimize the parameters of the network structure in order to obtain the desired optimum model. Once trained, the learned features can be used to classify new data. Unsupervised feature learning is the direct modeling of input data and combining data with a high level of similarity. The new data can then be identified by similarity calculation to determine which category it belongs to, thus achieving the goal of classification. Semisupervised feature learning is first learned with unsupervised feature learning and then supervised feature learning is used to improve the performance [13, 14]. Deep learning improves the efficiency of rolling bearing fault detection through iterative analysis of data. Deep learning models include convolutional neural networks, deep trust network models, and stack self-encoding network models. The deep learning model is shown in Figure 1.

The research directions of deep learning are as follows:

1. There are two purposes of speech recognition: the first is to recognize the syllables of each word in the speech. Then, the recognized syllables are formed into words according to the semantics. In China, Baidu and iFLYTEK have taken the lead in this field, taking the lead in breaking through key technologies. Baidu, in particular, still has 81% accuracy for speech recognition in very noisy environments. This result is far superior to other famous companies such as Google [15].
2. Natural language processing is a technology that enables people to communicate with computers directly through language. After years of development, deep learning has not developed very rapidly in this field. In the research, it was found that the processing ability of deep learning for natural language is not as strong as that in the field of speech and images. However, related technical research is still in progress, and it is believed that there will be a good development in the near future.
3. To date, deep learning has achieved very impressive results in the field of pattern recognition. Since 2012, different models have been proposed one after the other. The accuracy of image recognition is getting higher and higher. The application of deep learning is also very widespread. The accuracy of facial recognition in various competitions is constantly improving. In many companies, punching machines with facial recognition have replaced the original card swiping or fingerprint checking machines. Cars with automatic number plate recognition are also appearing in car parks. It is therefore believed that image recognition will be widely used in the future [16].

Deep learning is an internal rule and expression level for learning from sample data. The information gained during this learning process will greatly aid in understanding information such as words, images, and sounds. Deep learning is to learn the inherent laws and representation levels of sample data, and the information obtained during these learning processes is of great help to the interpretation of data such as text, images, and sounds [17].

The key to artificial intelligence lies in how to mimic the brain's ability to express information efficiently and accurately. Deep learning is more abstract in high-level elements that are made up of low-level elements to mimic the underlying structure of the brain. In the brain, perception of things occurs in layers, with edge features being extracted first from the most primitive data, then at the next layer and then at a higher level. Perception of the world in the brain is therefore a process of continuous abstraction, iteration, and learning of rules layer by layer. And these kinds of patterns can significantly reduce the amount of data the nervous system has to process and retain the most important information. The mechanism of the human brain is shown in Figure 2.

Rolling bearings are used in most rotating machines. They are widely used because they offer advantages such as high rotational efficiency, low power losses, and low starting friction torque. However, the mechanical structure of a rolling bearing results in a relative movement between the inner and outer ring when the bearing rotates. At the same time, the load is unevenly distributed on the rolling elements during the rotation of the bearing, so the rolling bearing is easily damaged during operation.

The failure forms of rolling bearings are mainly manifested in the following four aspects:

1. Fatigue failure: the main reason is that the rolling elements are repeatedly subjected to periodic loads on the raceway, which in turn causes the surface of the bearing to be subjected to alternating stress.
2. Wear failure: the main reason is the excessive friction between the ball and the raceway. For example, rolling bearings are often overloaded, bearing insufficient lubrication, improper assembly, etc. During the operation of the rolling bearing, foreign objects fall into the groove of the bearing, causing it to be worn and damaged.
3. Corrosion failure: the main reason is that the humidity in the air is too high or the operating environment contains corrosive media. Once the protection measures of the bearing are not comprehensive, electrochemical corrosion is prone to occur. This will eventually increase the corrosion of the bearing, which will lead to defects in the bearing surface and accelerate the failure of the bearing.
4. Fracture failure: the main reason is that the metal material of the bearing is insufficient, overload operation, and poor heat treatment. When the bearing breaks, it usually causes the equipment to stop running, and when the situation is serious, it will cause a large accident, which is very dangerous.

There are currently three main approaches to deep learning: the autoencoder (AE), the constrained Boltzmann machine (RBM), and the convolution neural network (CNN). However, since this paper only uses the autoencoder deep learning approach, only the autoencoder deep learning approach is presented here.

Self-encoding has evolved from neural networks and is the oldest deep learning method. The purpose of the autoencoder is to make the input and output as equal as possible, and adjust the network parameters through the residual between the input and output. The structure of the autoencoder is shown in Figure 3.

In the auto-encoding of the network, there are two steps. The process from the input layer to the hidden layer is called the encoding process. The process from the hidden layer to the output layer is called decoding. The original data is input into the encoder by the output layer, and the nonlinear transformation is performed to obtain the activation value of the hidden layer nodes.

In the traditional fault detection method, information can be hidden due to the influence of design parameters and it is not possible to extract all the information from the data. To extract more useful information from the data requires a more complex and deep network structure. Deep learning methods attempt to learn the deep nonlinear network structure, achieve a more complex feature approximation and learn more classifiable eigenvalues.

A stacked sparse autocoding network (SSAE) is constructed by stacking several autocoding networks. Therefore, the whole network can be trained by the layer-by-layer training method instead of training the whole network at once.  Figure 4 shows the structure of a self-coding network. The input data can be described in a higher dimensionality, which facilitates detection of information hidden in the input data. Stacking autoencoders can effectively extract data features, but they have poor generalization and are not suitable for network fluctuation data traffic. On the basis of the single-layer sparse autoencoder, adding sparse constraints can effectively reduce the trained overfitting problem.

The function of the autoencoder is to learn the representation of the input information by taking the input information as the learning target. After layer-by-layer training, all parameters of each layer of the entire network can be adjusted to the best. But in the process of training each layer, other layers are fixed. It is impossible for the residual to reach 0 during training, so after layer-by-layer training, the residual of the previous layer will always propagate backwards. In the end it will lead to unsatisfactory results. Since each layer of the network has been pretrained, the adjustment in this global training is relatively small, so it is called global fine-tuning. Fine-tuning reduces errors due to residual propagation and also avoids local optima caused by directly training the entire network.

The basic idea of rolling bearing fault detection based on stacked sparse self-encoding: the first is to process the raw data to create the required training and test set. Then, we train the entire network using the training set. During training, the network is trained layer by layer using the unsupervised method, and then fine-tuned using the supervised method. Finally, the performance of the whole network is verified using a test set for fault detection. The deep learning based fault detection consists of three parts: preprocessing module, deep learning module, and fault detection module. The idea of the fault detection module is similar to that of pattern recognition and aims to classify the input data.  Figure 5 shows a block diagram of rolling bearing fault detection based on stacked sparse self-coding, which contains two self-coding hidden layers.

Although SSAE can significantly improve the efficiency of rolling bearing defect detection, the results are not satisfactory. The reason is that the layers are completely connected and the network has too many parameters. This creates too much complexity and is easily overestimated during training. At the same time, the correlation between distant points is weak or even negligible. However, full connectivity will result in some correlation between these remote points. Although this correlation may be weak, it will have more or less influence. If the similarity between two points that are far apart is relatively large, then there should be no correlation between them because of the relatively large distance. But this may also eventually lead to the network learning strong correlations.

For the logistic regression algorithm, the goal is to get a 0/1 model that maps the independent variables to 0, 1 when used. The mapped value is the probability that *y* = 1. Its formal function is expressed as

(1) $$\begin{array}{c} h_{\theta }\left(x\right)=\frac{1}{1+e^{{-\theta }^{T}x}}\text{.} \end{array}$$

As shown in Figure 6, the purpose of the logistic regression algorithm is to find the middle line, so that different types of data are distributed on both sides of the line, and all points are as far away from the line as possible. Supposing there are two points A and B, and B belongs to class ×. But the distance between A and the straight line is relatively close. It ensures that both A and B fall into the category × area by keeping A as far away from the line as possible. Therefore, only the distance between point A and the line needs to be considered here, not A and B and other points further apart. This makes it possible to consider only a part of the points that have an impact on the results, not all of them, when learning the model, which is the basic idea of SVM.

In SVM, the labels of the output results use *y* = −1 and *y* = 1. At the same time, let *θ*^*T*^*x*=*w*^*T*^*x*+*b*, we get

(2) $$\begin{array}{c} h_{\theta }\left(x\right)=g\left(\theta^{T}x\right)=g\left(w^{T}x+b\right)\text{.} \end{array}$$

Since the result of formula (1) is only related to the positive and negative of *θ*^*T*^*x*, and there is no need to consider *g*(*x*), *g*(*x*) can be simplified as follows:

(3) $$\begin{array}{c} g\left(x\right)=sign\left(x\right)=\left\{\begin{array}{cc} 1 & ,x\geq 0\text{,}\\ -1 & ,x<0\text{.} \end{array}\right. \end{array}$$

(4) $$\begin{array}{c} \frac{y^{\left(i\right)}}{\left\|w\right\|}=\frac{\left(w^{T}x^{\left(i\right)}+b\right)}{\left\|w\right\|}\text{.} \end{array}$$

Then, the distance of (*w*^*T*^*x*^(*i*)^+*b*) is called the function distance. Formula (4) is the geometric distance. Therefore, when *w* and *b* are expanded by the same times, the function distance is expanded by the same times, but the geometric distance remains unchanged, and when ‖*w*‖, the functional distance and the geometric distance are equal.

(5) $$\begin{array}{c} \min_{x^{\left(i\right)}}\frac{\left\|w^{T}x+b\right\|}{\left\|w\right\|}\text{.} \end{array}$$

The final formula to be optimized is

(6) $$\begin{array}{c} \max_{w,b}\left[\min_{x^{\left(i\right)}}\frac{y^{\left(i\right)}\left(w^{T}x+b\right)}{\left\|w\right\|}\right]\text{,} \end{array}$$

when *w* and *b* increase by the same fold, the geometric distance does not change. But what is needed here are definite values of *w* and *b*, and not multiples of them. Therefore, it is necessary to add constraints to it to ensure the uniqueness of the solution. For simplicity, let *y*^(*i*)^(*w*^*T*^*x*+*b*)=1, so that the global function interval can be defined as 1. Then the distance from the closest point to the hyperplane is (1/‖*w*‖), so formula (6) can be transformed into

(7) $$\begin{array}{c} \max_{w,b}\frac{1}{\left\|w\right\|}\text{.} \end{array}$$

(8) $$\begin{array}{c} \min_{w,b}\frac{1}{2}{\left\|w\right\|}^{2}\text{.} \end{array}$$

To optimize formula (8), it is transformed here using Lagrangian formula and KTT condition as follows:

(9) $$\begin{array}{c} \min_{w,b}\max_{\alpha }L\left(w,b,\alpha \right)\text{.} \end{array}$$

Among them,

(10) $$\begin{array}{c} \max_{\alpha }L\left(w,b,\alpha \right)=\frac{1}{2}{\left\|w\right\|}^{2}-\overset{m}{\underset{i=1}{\sum }}\alpha_{i}\text{.} \end{array}$$

According to the duality principle, we get

(11) $$\begin{array}{c} \max_{\alpha }\min_{w,b}L\left(w,b,\alpha \right)=\min_{w,b}\max_{\alpha }L\left(w,b,\alpha \right)\text{.} \end{array}$$

(12) $$\begin{array}{c} \frac{\partial L\left(w,b,\alpha \right)}{\partial w}=w-\overset{m}{\underset{i=1}{\sum }}\alpha_{i}y\text{.} \end{array}$$

(13) $$\begin{array}{c} \frac{\partial L\left(w,b,\alpha \right)}{\partial b}=\overset{m}{\underset{i=1}{\sum }}\alpha_{i}\text{.} \end{array}$$

From formula (12), we get

(14) $$\begin{array}{c} w=\overset{m}{\underset{i=1}{\sum }}\alpha_{i}y\text{.} \end{array}$$

Bringing formula (13) and formula (14) into *L*(*w*, *b*, *α*) gives

(15) $$\begin{array}{c} L\left(w,b,\alpha \right)=\overset{m}{\underset{i=1}{\sum }}\alpha_{i}-\frac{1}{2}\overset{m}{\underset{i=1}{\sum }}\alpha_{j}y_{i}\text{,}\\ \alpha^{*}=arg\max_{\alpha }\left(\overset{m}{\underset{i=1}{\sum }}\alpha_{i}-\frac{1}{2}\overset{m}{\underset{i=1}{\sum }}\overset{m}{\underset{j=1}{\sum }}\alpha_{i}\alpha_{j}y_{i}y_{j}\right)\text{.} \end{array}$$

Thus, we get

(16) $$\begin{array}{c} w^{*}=\overset{m}{\underset{i=1}{\sum }}\alpha_{i}^{*}y\text{,}\\ b^{*}=y_{i}-\overset{m}{\underset{i=1}{\sum }}\alpha_{i}^{*}y_{i}\langle x_{i},x_{j}\rangle \text{.} \end{array}$$

The optimal splitting hyperplane is

(17) $$\begin{array}{c} w^{*}x^{\left(i\right)}+b^{*}=0\text{.} \end{array}$$

The final decision function is

(18) $$\begin{array}{c} f\left(x\right)=sign\left(w^{*}x_{i}+b^{*}\right)\text{.} \end{array}$$

In this paper, the features of the support vector machine (SVM) classifier algorithm are used to detect rolling bearing defects for the purpose of eliminating bearing defects.

## 3. Rolling Bearing Fault Detection Experiment

The design parameters of the rolling bearing are shown in Table 1.

Bearing data for the drive end of the test bench are shown in Tables 2 and 3.

The data provided by the experiment are time series signals and therefore cannot be used directly. At the time of data acquisition, the bearing speed was 1797 r/min. The sensors used to collect signals can collect 12,000 signals per second. Therefore, it can be obtained that about 400 signals can be collected for each rotation of the bearing. Therefore, 400 consecutive signals can be defined as one sample data. This gives us a useable training and test set from the original data. A total of 600 samples of normal signals and 300 samples of faulty signals were obtained in this experiment.

The softmax classifier is first trained on training samples and then its performance is tested on test samples. The overall correct rate is 70.571%, and the correct rate for each data type is shown in Figure 7(a). The classification accuracy of the SVM classifier for each data type is shown in Figure 7(b).

Figure 7(a) shows that the softmax classifier has a high detection rate for normal signals. But the fault signal is very poor, and the false alarm rate is high. Although the normal signal can be judged, the judgment result for the fault signal is very poor, so the overall effect is relatively poor. Figure 7(b) shows that the SVM classifier achieves 100% classification accuracy for normal signals, which is higher than the classification accuracy of other data types.

Figure 8 shows the results for different numbers of nodes in the hidden layer. For the classification accuracy of the number of nodes in different hidden layers, the first is an upward trend, the next is a downward trend, and the overall stability is relatively stable.

Figure 8 shows that with different number of nodes, the entire model has different classification accuracy on the test set. It also shows that the number of hidden layer nodes has no significant relationship with the classification accuracy.

To investigate the effect of the number of network layers on its performance, a third SAE network structure is added on this basis. It sets the number of hidden layer nodes to 600, 400, and 200 sequentially, and sets the number of iterations to 400. Its overall correct rate is 88.571%. The correct rate of each data type is shown in Figure 9.

Figure 9 shows that SSAE classification accuracy does not increase with the number of layers. Since the training data set is limited, adding more hidden layers increases the number of parameters. This increases the complexity of the network. If the training set is fixed and the number of samples is not very large, the results often do not improve significantly. It may even make the results worse if the network parameters are increased. In an experiment, since the initial value of the network is generated randomly in each simulation, there will be some bias in the results of each simulation. Therefore, the final accuracy did not increase, but it did not decrease significantly either. This suggests that increasing the number of layers in the network can no longer improve the overall network performance, but it currently has no effect on the network performance. However, if hidden layers continue to be added, the overall performance may decrease due to an increase in network parameters. Therefore, the following experiments use a network structure with two hidden layers.

Tables 4 and 5 present the results of specific solutions for each data type. For simplicity, labels are used to denote error types. The last row indicates the number of samples for each data type in the test set. Each row indicates the number of samples corresponding to the data type evaluated in the column corresponding to the row. For example, 8 in the fifth row of the third column indicates that the failure of data type 3 is judged as the number of failures of data type 5 is 8.

Tables 4 and 5 show that the SVM classifier can detect all the faults and also does not judge the faulty signal as a normal signal. But the detection of faults is not very accurate. Especially for the outer ring failure, the misjudgment rate is very high. Therefore, using this method directly can be used for fault detection, but it cannot be used for fault detection. The SVM classifier can be combined with other classification detection methods for experimental analysis.

Figure 10 shows the detection accuracy of four classifiers: softmax, KNN, Bayes, and SVM, on the original data and the detection accuracy after combining with the three networks, respectively.

Figure 10 shows that the three grid structures have improved the accuracy of rolling bearing defect detection. The performance improvement is particularly evident, especially when combined with the softmax classifier and the SVM classifier. Compared to an ordered autoencoder grid, the local map autoencoder grid and the local loop map autoencoder grid have a negligible effect on the improved defect detection performance of the softmax classifier. However, it still has some effect on the fault detection performance of the SVM classifier. The performance of the local recurrent map autoencoder is higher than that of the local map autoencoder. But this impact is not very large. This is due to the fact that the dimensionality of each sample of the dataset used in the experiments is 400. In local connectivity, each node of the input layer is connected to only 5 nodes of the hidden layer. Then, only 3 nodes of the hidden layer are touched in the network in order to obtain correlation between the head node and the back node and to adopt local cyclic mapping. After calculations, it can be concluded that there are 800 nodes in the hidden layer, so the affected nodes are only 0.375% of the total. However, this also increased the detection accuracy by 0.6 percentage points. This also proves that this method is suitable for detecting rolling bearing defects. Softmax classifier and SVM classifier combined with deep learning can improve the efficiency of rolling bearing fault detection.

## 4. Discussion

Deep learning enables computers to simulate human vision, thinking, and other behaviors and solve a large number of complex pattern recognition problems. Deep learning has made a lot of achievements in search technology, data mining, machine learning, machine translation, natural language processing, multimedia learning, speech, recommendation and personalization technology, and other related fields. It is a bold attempt to introduce deep learning into the paper.

At present, the research on rolling bearings in the field of fault detection is roughly in the following three directions.

### 4.1. Integration of Signal Processing Technologies

The cause of equipment failure is usually not a single factor, or multiple points of failure. Traditional detection methods use only a single signal processing method. This fault detection technique is targeted. When dealing with the faults of different workpieces, this method often cannot achieve better processing results. At present, the detection methods of rolling bearings are moving towards the fusion of multisignal analysis methods. The fusion of multiple signal processing technologies can show their respective strengths and can usually achieve the expected processing effect obviously.

### 4.2. Integrate Nonlinear Theory

Rolling bearing fault signals are usually nonlinear. At present, there are certain limitations for nonlinear processing methods, for example, Lyapunov method, phase plane method, and description function method. Therefore, the integration of nonlinear theory research and rolling bearing fault detection will bring bearing fault detection to a new level.

### 4.3. Fusion of Modern Signal Analysis Methods and Intelligent Detection

At present, intelligent detection technology is also developing rapidly, for example, algorithms such as evolutionary computing, genetic algorithm, and neural network. The fusion of these algorithms with modern signal processing methods has gradually become closer and the application has become very extensive. New scientific research technology can usually drive the rapid development of a certain research field and the continuous progress of science and technology. Intelligent detection technology will have broad prospects for development.

## 5. Conclusion

Rolling bearing damage is different from ordinary damage. Rolling bearings have their own periodic characteristics, so special attention must be paid to this characteristic. (1) This paper describes rolling bearing fault detection based on SSAE. This method examines features from raw data using SSAE. It is then classified, i.e., fault detection is performed. The network parameters are optimized using a training set to optimize the network performance. After the sample data passes through the network, an abstract representation of the sample is obtained, which improves the detection accuracy. (2) Local sampling can be achieved by autocoding with local mapping, but the original periodicity of the signal is lost. This impairs the detection result. Based on rolling bearing periodicity, a local autocoder with cyclic mapping is proposed in this paper. The nodes in each layer of the network are connected to each other. Thus, the sampling data is circular and the correlation between the head and tail nodes will not be lost. The experiments investigate all classification problems, including classification between defects and normal data as well as classification between defects. However, the correlation between different levels of the same defect has not been investigated. Therefore, further research on defect severity is needed in future work.

## Figures and Tables

**Figure 1:** Deep learning model.

**Figure 2:** Human brain mechanism.

**Figure 3:** Self-encoding network structure.

**Figure 4:** Autoencoding network.

**Figure 5:** Rolling bearing fault detection process based on stacked sparse self-encoding.

**Figure 6:** Logistic regression algorithm model.

**Figure 7:** Classification accuracy of different classifiers for each data type. (a) Type Of data. (b) Type of data.

**Figure 8:** Classification accuracy with different number of hidden layer nodes.

**Figure 9:** Classification accuracy of softmax classifier after SSAAE learning with different layers. (a) Type of data. (b) Type of data.

**Figure 10:** Detection accuracy of different classifiers combined with different network structures. (a) Classifier. (b) Classifier.

**Table 1:** Rolling bearing structural parameters.

Inner ring	Outer ring diameter	Rolling body	Thickness
25 mm	52 mm	8mm	15 mm
Diameter	Contact angle	Number of balls	Bearing speed
39 mm	0 degree	8	1797 rpm

**Table 2:** Bearing data of the drive end part of the test bench.

Data set	Condition	Damage scale/mm	Label
A	Normal	—	1
	Ball failure	0.1778	2
	Inner ring failure	0.1778	3

**Table 3:** Bearing data of the drive end part of the test bench.

Data set	Condition	Damage scale/mm	Label
B	Outer ring failure at three o'clock	0.1547	4
	Outer ring failure at six o'clock	0.4128	5
	Twelve o'clock fault of outer ring	0.5334	6

**Table 4:** SVM classifier judgment results for each kind of data.

Type of data	1	2	3	4	5	6
1	200	0	0	0	0	0
2	0	74	2	4	36	45
3	0	0	90	30	0	0

**Table 5:** SVM classifier for each kind of data decision results.

Type of data	1	2	3	4	5	6
4	0	0	0	64	0	0
5	0	7	8	2	56	3
6	0	19	0	0	8	52

## Data Availability

The data used to support the findings of this study are available from the author upon request.
